The article "Prevalence and clinical features of hearing loss caused by EYA4 variants" was published in 2020. Journal: Sci Rep.

# Prevalence and clinical features of hearing loss caused by *EYA4* variants

**DOI:** 10.1038/s41598-020-60259-0

**Published:** 2020-02-27

**Authors:** Jun Shinagawa, Hideaki Moteki, Shin-ya Nishio, Kenji Ohyama, Koshi Otsuki, Satoshi Iwasaki, Shin Masuda, Chie Oshikawa, Yumi Ohta, Yasuhiro Arai, Masahiro Takahashi, Naoko Sakuma, Satoko Abe, Yuika Sakurai, Hirofumi Sakaguchi, Takashi Ishino, Natsumi Uehara, Shin-ichi Usami

**Affiliations:** 1 Department of Otorhinolaryngology, Shinshu University School of Medicine, 3-1-1 Asahi, Matsumoto, Nagano 390-8621 Japan; 2 Department of Hearing Implant Sciences, Shinshu University School of Medicine, 3-1-1 Asahi, Matsumoto, Nagano 390-8621 Japan; 3 Department of Otolaryngology, Tohoku Rosai Hospital, 4-3-21 Dainohara, Aoba-ku, Sendai, Miyagi 981-8563 Japan; 4 Department of Otolaryngology, Fukushima Medical University, 1 Hikariga-oka, Fukushima, Fukushima 960-1295 Japan; 5 Department of Otorhinolaryngology, International University of Health and Welfare, Mita Hospital, 1-4-3 Mita, Minato-ku, Tokyo 108-8329 Japan; 6 Department of Pediatric Rehabilitation, Hiroshima Prefectural Hospital, 1-5-54 Ujina-Kanda, Minami, Hiroshima 734-8530 Japan; 7 Department of Otorhinolaryngology and Head and Neck Surgery, Graduate School of Medical Sciences, Kyushu University, 3-1-1, Maidashi, Higashi-ku, Fukuoka, Fukuoka 812-8582 Japan; 8 Department of Otorhinolaryngology-Head and Neck Surgery, Graduate School of Medicine, Osaka University, 2-2 Yamadaoka, Suita, Osaka 565-0871 Japan; 9 Department of Otorhinolaryngology, Head and Neck Surgery, Yokohama City University School of Medicine, 3-9 Fukuura, Kanazawa-ku, Yokohama, Kanagawa 236-0004 Japan; 10 Department of Otorhinolaryngology, Yokohama City University Medical Center, 4-57 Urafune, Minami-ku, Yokohama, Kanagawa 232-0024 Japan; 11 Department of Otorhinolaryngology, Toranomon Hospital, 1-2-3 Toranomon, Minato-ku, Tokyo 105-0001 Japan; 12 Department of Otorhinolaryngology, Jikei University School of Medicine, 3-25-8 Nishi-Shimbashi, Minato-ku, Tokyo 105-8461 Japan; 13 Department of Otorhinolaryngology-Head and Neck Surgery, Kyoto Prefectural University of Medicine, Kawaramachi-Hirokoji, Kajii-cho, Kamigyo-ku, Kyoto, Kyoto, 602-8566 Japan; 14 Department of Otorhinolaryngology, Head and Neck Surgery, Graduate School of Biomedical and Health Sciences, Hiroshima University, 1-2-3 Kasumi, Minami-ku, Hiroshima, Hiroshima, 734-8553 Japan; 15 Department of Otorhinolaryngology, Head and Neck Surgery, Kobe University School of Medicine, 7-5-1 Kusunoki-machi, Chuou-ku, Kobe 650-0017 Japan

**Keywords:** Genetic testing, Genetics research

## Abstract

Variants in the *EYA4* gene are known to lead to autosomal dominant non-syndromic hereditary hearing loss, DFNA10. To date, 30 variants have been shown to be responsible for hearing loss in a diverse set of nationalities. To better understand the clinical characteristics and prevalence of DFNA10, we performed genetic screening for *EYA4* mutations in a large cohort of Japanese hearing loss patients. We selected 1,336 autosomal dominant hearing loss patients among 7,408 unrelated Japanese hearing loss probands and performed targeted genome enrichment and massively parallel sequencing of 68 target genes for all patients. Clinical information of cases with mutations in *EYA4* was gathered and analyzed from medical charts. Eleven novel *EYA4* variants (three frameshift variants, three missense variants, two nonsense variants, one splicing variant, and two single-copy number losses) and two previously reported variants were found in 12 probands (0.90%) among the 1,336 autosomal dominant hearing loss families. The audiometric configuration of truncating variants tends to deteriorate for all frequencies, whereas that of non-truncating variants tends to show high-frequency hearing loss, suggesting a new correlation between genotype and phenotype in DFNA10. The rate of hearing loss progression caused by *EYA4* variants was considered to be 0.63 dB/year, as found in this study and previous reports.

The article "Prevalence and clinical features of hearing loss caused by EYA4 variants" was published in 2020. Journal: Sci Rep.

## Introduction

Hearing loss is the most common sensory disorder and more than 50% of cases of congenital or early onset hearing loss are caused by genetic factors^1^. Regarding hereditary hearing loss, over 100 genes are known to be causative based on genetic analysis [Hereditary Hearing Loss Homepage: https://hereditaryhearingloss.org/ accessed at August 2019], and this identification has been accelerated by the recent progress in genome sequencing technology. Hereditary hearing loss patterns vary between autosomal dominant, autosomal recessive, X-linked, and mitochondrial. Autosomal dominant non-syndromic hearing loss (ADNSHL) is often seen in postlingual hearing loss patients, and is the cause for approximately 20–25% of all hereditary hearing loss^2^. Currently, 67 causative genes for ADNSHL have been identified^3^.

The *EYA4* gene (OMIM* 603550), located on chromosome 6q22.3-q23.2, for DFNA10 (OMIM# 601316) was first identified in American and Belgian hearing loss patients in 2001^4^. *EYA4* encodes eye absent 4 protein, a member of the EYA family of proteins. It is a transcriptional activator and is considered to be required for proper eye development as well as for the maturation and maintenance of the organ of Corti^5^. It has been reported that *Eya4* is expressed in early stage otic vesicles, largely confined to the upper cochlear duct, in rodents. These cells later form the stria vascularis, Reissner’s membrane, spiral limbus, and organ of Corti. *Eya4* is also expressed in the spiral ganglion neurons and organ of Corti in marmosets; however, the expression pattern in the human cochlea remains unknown^6^. The EYA4 protein is comprised of 639 amino acids with 2 functional domains. The C-terminal domain, which is composed of 271 residues and is named eyaHR (alternatively called the eya domain or eya homology domain 1), is highly conserved among EYA family proteins, and a more divergent proline-serine-threonine (PST)-rich transactivation domain is located at the N-terminus (eyaVR).

The article "Prevalence and clinical features of hearing loss caused by EYA4 variants" was published in 2020. Journal: Sci Rep.

To date, 30 variants in the *EYA4* gene and a partial or whole deletion of the *EYA4* allele have been reported as a cause of ADNSHL in various ethnic groups, including the American, Belgian, Dutch, Korean, Chinese, Swedish, German, Australian, Hungarian, Philippine, Italian, and Japanese populations^4,5,7–31^. These previous studies have described the clinical phenotypes of patients with *EYA4* variants; however, the detailed characteristics of the hearing loss, such as its progressiveness or severity, remain unclear. In addition, the genotype-phenotype correlation is also yet to be clarified.

In this study, we sought to elucidate the variant spectrum of the *EYA4* gene and prevalence of *EYA4-*associated hearing loss in the Japanese population, and to obtain a more precise description of the clinical features of *EYA4-*associated hearing loss.

## Materials and Methods

### Study subjects

A total of 7,408 probands from unrelated Japanese hearing loss families were enrolled from 67 otolaryngology departments across Japan participating in the present study between February 2012 and October 2017. The hereditary patterns of the hearing loss in the probands’ families were autosomal dominant in 1,336, autosomal recessive/sporadic in 4,898, and unknown inheritance pattern in 1,174 cases. Written informed consent was obtained from all patients (or from their next of kin, caretaker, or legal guardian in case of minors or children). This study was approved by the Shinshu University Ethical Committee as well as the respective Ethical Committees of the other participating institutions listed below. Akita University Ethical Committee, Iwate Medical University Ethical Committee, Tohoku Rosai Hospital Ethical Committee, Fukushima Medical University Ethical Committee, Yamagata University Ethical Committee, Dokkyo Medical University Ethical Committee, TAKASAKI Ear Nose & Throat Clinic Ethical Committee, Niigata University Ethical Committee, Tokyo Medical University Ethical Committee, Jikei University Ethical Committee, Toranomon Hospital Ethical Committee, Kitasato University Ethical Committee, International University of Health and Welfare Mita Hospital Ethical Committee, National Rehabilitation Center for Persons with Disabilities Ethical Committee, Keio University Ethical Committee, Hamamatsu University Ethical Committee, Shiga University Ethical Committee, Shiga Medical Center for Children Ethical Committee, Osaka University Ethical Committee, Kobe City Medical Center General Hospital Ethical Committee, Hyogo College of Medicine Ethical Committee, Kyoto Prefectural University Ethical Committee, Okayama University Ethical Committee, Yamaguchi University Ethical Committee, Ehime University Ethical Committee, Kyushu University Ethical Committee, Kanda ENT Clinic Ethical Committee, Nagasaki University Ethical Committee, Miyazaki University Ethical Committee, Kagoshima University Ethical Committee, Ryukyus University Ethical Committee, Sapporo Medical University Ethical Committee, Tohoku University Ethical Committee, Jichi Medical University Ethical Committee, Gunma University Ethical Committee, Jyuntendo University Ethical Committee, Yokohama City University Ethical Committee, Mejiro University Ethical Committee, Saitama Medical University Ethical Committee, Abe ENT clinic Ethical Committee, Tokyo Medical Center Institute of Sensory Organs Ethical Committee, Jichi University Saitama Medical Center Ethical Committee, Aichi Children’s Health Medical Center Ethical Committee, Chubu Rosai Hospital Ethical Committee, Kyoto University Ethical Committee, Mie University Ethical Committee, Kansai Medical University Ethical Committee, Kobe University Ethical Committee, Osaka Medical Center and Research Institute for Maternal and Children Health Ethical Committee, Wakayama Medical University Ethical Committee, Kouchi University Ethical Committee, Hiroshima University Ethical Committee, Hiroshima City Hiroshima Citizen Hospital Ethical Committee, Fukuoka University Ethical Committee, Kurume University Ethical Committee, National Defense Medical College Ethical Committee, Tokai University Ethical Committee, Hokkaido University Ethical Committee, Kanagawa Children’s Medical Center Ethical Committee, Tokyo Medical and Dental University Ethical Committee, Hirosaki University Ethical Committee, Tokyo Metropolitan Children’s Medical Center Ethical Committee, Hakodate central general hospital Ethical Committee, Osaka Red Cross Hospital Ethical Committee, Hiroshima Prefectural Hospital Ethical Committee, Nara Medical University Ethical Committee, and Tsukuba University Ethical Committee. All methods were performed in accordance with the Guidelines for Genetic Tests and Diagnoses in Medical Practice of the Japanese Association of Medical Sciences and the Declaration of Helsinki as required by Shinshu University.

The article "Prevalence and clinical features of hearing loss caused by EYA4 variants" was published in 2020. Journal: Sci Rep.

### Clinical evaluations

The onset age of hearing loss and the degree of progressiveness were analyzed based on the medical charts of the probands and their family members harboring the same *EYA4* variants. Pure-tone average (PTA) was calculated from the audiometric thresholds at four frequencies (0.5, 1, 2, and 4 kHz). The severity of hearing loss was divided into mild (PTA: 20–40 dB HL), moderate (41–70 dB HL), severe (71–95 dB HL), and profound (>95 dB HL). Asymmetric hearing loss was defined as a difference in PTA of over 10 dB between the right and left ears. The audiometric configurations were categorized into low-frequency, mid-frequency (U-shaped), high-frequency, flat type, and deaf as reported previously^32^.

### Amplicon resequencing and variant annotation

Amplicon libraries were prepared using an Ion AmpliSeq™ Custom Panel for 68 genes reported to cause non-syndromic hereditary hearing loss (ThermoFisher Scientific, MA, USA), in accordance with the manufacturer’s instructions. The detailed protocol has been described elsewhere^33^. MPS was performed with an Ion Torrent Personal Genome Machine (PGM) system using an Ion PGM™ 200 Sequencing Kit and an Ion 318™ Chip (ThermoFisher Scientific). The sequence data were mapped against the human genome sequence (build GRCh37/hg19) with a Torrent Mapping Alignment Program. After sequence mapping, the DNA variant regions were piled up with Torrent Variant Caller plug-in software. After variant detection, their effects were analyzed using ANNOVAR software^34,35^. The missense, nonsense, insertion/deletion and splicing variants were selected from among the identified variants. Variants were further selected as less than 1% of: (1) the 1,000 genome database, (2) 6,500 exome variants, (3) the Human Genetic Variation Database (a dataset for 1,208 Japanese exome variants), and (4) 333 in-house Japanese normal hearing controls. This filtering process was performed using our original database software described elsewhere^36^. The pathogenicity of selected variants was evaluated by ACMG (American College of Medical Genetics) standards and guidelines^37^. For missense variants in particular, functional prediction software, including Sorting Intolerant from Tolerant (SIFT), Polymorphism Phenotyping (PolyPhen2), LRT, Mutation Taster, Mutation Assessor, Functional Analysis through Hidden Markov Models (FATHMM), RadialSVM, LR, and CADD, were used through the ANNOVAR software program^34,35^. Direct sequencing was utilized to confirm the selected variants.

The article "Prevalence and clinical features of hearing loss caused by EYA4 variants" was published in 2020. Journal: Sci Rep.

### Copy number analysis in the MPS database

We employed our recently published specialized copy number variation (CNV) detection method for Ion AmpliSeq^TM^ sequencing that utilizes multiplex PCR-based targeted genome enrichment^38^. The depth of coverage information for each amplicon was used for copy number analysis. After normalization, the relative read depths of amplicons were visualized as described previously^38^.

### Variant prioritization

*EYA4* was reported as a genetic cause for autosomal dominant inherited hearing loss, thus, we selected hearing loss patients from apparently autosomal dominant families. Among 1,336 autosomal dominant hearing loss families, we further selected the families with candidate *EYA4* variants. The criteria for the selection process were (1) the *EYA4* variant was classified into “pathogenic”, “likely pathogenic” or “uncertain significance” and (2) there were no candidate variants in the other 67 genes reported to cause hearing loss. Based on the ACMG guidelines, we regarded “pathogenic” and “likely pathogenic” variants as strong candidates for *EYA4*-associated hearing loss. In addition, we listed the “variants of uncertain significance” identified during the filtering procedure described above in Table 1. However, we removed “variants of uncertain significance” with a CADD Phred score of less than 20, or identified in some control databases as being of “unlikely causative”. The CADD Phred score threshold used in this study was <20 as all of the previously reported *EYA4* pathogenic variants were predicted to have a CADD Phred score of 23.5 or more (e.g., the lowest CADD Phred score for c.978C > G is 23.5), so we employed 20 as threshold to allow a safety margin. In addition, we also removed the c.1790delT and c.1886_1899del variants as unlikely causative variants because nonsense-mediated mRNA decay was not presumed to be triggered from the location of the variants. Finally, we selected 12 variants as causative and performed a more detailed hearing loss phenotype analysis.

**Table 1:** All *EYA4* variants found in this study.

#	RefSeq ID	Nucleotide Change	Amino Acid Change	Exon	Domain	Genomic position (GRCh37.p5)	SIFT	PolyPhen2_HVIR	PolyPhen2_HVAR	LRT	Mut _Taster	Mut _Assessor	FATHMM	Meta SVM	Meta LR	CADD_Phred	Allele Frequency (Exac03)		ACMG criteria (supporting evidence)
Likely causative																			
1	NM_004100	c.222_223del	p.T74fs	5	V	133769262											0		Likely Pathogenic (PVS1 + PM2)
2	NM_004100	c.498delG	p.Q166fs	8	V	133783533											0		Likely Pathogenic (PVS1 + PM2)
3	NM_004100	c.517C > T	p.Q173X	8	V	133783552				0.843	0.810					39.000	0		Likely Pathogenic (PVS1 + PM2 + PP3)
4	NM_004100	c.580 + 1G > A		intron 8	V	133783616					0.810					26.200	0		Likely pathogenic(PVS1 + PM2 + PP3)
5	NM_004100	c.910delC	p.P304fs	11	V	133789809											0		Likely Pathogenic (PVS1 + PM2)
6	NM_004100	c.988C > T	p.Q330X	12	V	133802618				0.843	0.810					47.000	0		Likely Pathogenic (PVS1 + PM2 + PP3)
7	NM_004100	c.1109G > C	p.R370P	13	E	133804171	0.912	0.899	0.971	0.629	0.810	0.888	0.975	0.995	0.984	34.000	0		VUS (PM2 + PP3)
8	NM_004100	c.1177C > T	p.Q393X	13	E	133804239				0.843	0.810					46.000	0.000008253	0.00009639(AFR)	Pathogenic (PVS1 + PS1 + PP3)
9	NM_004100	c.1216G > C	p.G406R	14	E	133827268	0.912	0.764	0.693	0.629	0.810	0.907	0.808	0.897	0.885	29.800	0		VUS (PM2 + PP3)
10	NM_004100	c.1663G > C	p.A555P	18	E	133844240	0.784	0.899	0.916	0.843	0.810	0.865	0.975	0.989	0.985	32.000	0		VUS (PM2 + PP3)
11	NM_004100			CNV		133782193–133789881													Likely pathogenic (PVS1 + PM2)
12	NM_004100			CNV		133756417–133852199													Likely pathogenic (PVS1 + PM2)
Unlikely causative																			
13	NM_004100	c.278T > C	p.M93T	6	V	133777694	0.153	0.090	0.127	0.305	0.810	0.065	0.623	0.514	0.500	14.76 *	0		VUS (PM2)
14	NM_004100	c.887C > T	p.S296L	11	V	133789786	0.721	0.548	0.533	0.629	0.537	0.741	0.853	0.816	0.812	23.600	0.00001651 **	0.0002(EAS) **	VUS (PP3)
15	NM_004100	c.936G > T	p.L312F	11	V	133789835	0.491	0.764	0.764	0.843	0.810	0.805	0.862	0.800	0.842	23.000	0.00001651 **	0.0002(EAS) **	VUS (PP3)
16	NM_004100	c.995C > T	p.P332L	12	V	133802625	0.348	0.764	0.739	0.843	0.810	0.684	0.953	0.970	0.972	27.900	0.000008264 **	0.0001(EAS) **	VUS (PS1 + PP3)
17	NM_004100	c.1790delT	p.V597fs	19	E	133846343											0		Pathogenic (PVS1 *** + PS1 + PM2)
18	NM_004100	c.1886_1899del	p.A629fs	20	E	133849909											0		VUS (PVS1 *** + PM2)

Abbreviation: V, variable region; E, Eya domain.

The article "Prevalence and clinical features of hearing loss caused by EYA4 variants" was published in 2020. Journal: Sci Rep.

*CADD score is low.

**MAF is too high.

***These variants are unlikely causative because nonsense-mediated mRNA decay is not presumed to be triggered from the location of the variants (see Discussion section).

## Results

### Identified variants and the frequency of EYA4-associated hearing loss

Among the 1,336 probands with ADNSHL, we identified 12 (0.90%) who carried a possible *EYA4* pathogenic variant (Table 1, Fig. 1). These 12 probands did not show any pathogenic variants or candidate variants in the 67 previously reported deafness genes apart from *EYA4*. Among the 12 candidate variants, eleven were novel, and one was previously reported. Three of them were missense variants, three were frameshift insertion/deletion variants, three were nonsense variants, one was a splicing variant, and two were copy number losses. Six of them were located in the eyaVR (amino acids 0–369) and four were located in eyaHR (amino acids 370–639). The one previously reported variant was classified as “Pathogenic”. Eight variants were classified as “Likely pathogenic” according to the ACMG guidelines, whereas three remained as “variants of uncertain significance (VUS)”. Further, none of the 12 variants was found in the Japanese 333 in-house controls (666 control alleles), and none of the three VUS variants was observed in the ExAC03 database.

**Figure 1:** Pedigrees and audiograms of twelve families who carried a possible *EYA4* pathogenic variant identified in this study. Filled symbols indicate affected individuals. Arrows indicate probands in each family. Unfortunately, we could not obtain DNA samples from family members except #12, so we could not perform family segregation analysis.

In addition to the above 12 causative *EYA4* variants, we also identified 6 variants in the *EYA4* gene from our cohort (Table 1), but we regarded these 6 variants as unlikely to be causative. Three missense variants, c.887C > T, c.936G > T, and c.995C > T were identified in the ExAC03 database over 0.0001, suggesting these three variants were not causative variants. In addition, the c.278T > C variant was predicted to be an unlikely causative variant from its low CADD score (CADD Phred score 14.76). Furthermore, the c.1790delT and c.1886_1899del variants were regarded as unlikely causative variants as nonsense-mediated mRNA decay was not presumed to be triggered from the location of the variants (these variants were located in the final exon or one exon before the final exon). From these results, the pathogenicity of these six variants was unclear. Thus, we performed further detailed clinical characteristic analysis for 12 patients with causative *EYA4* variants.

### Clinical characteristics of the EYA4-associated hearing loss patients identified in this study

Table 2 summarizes the clinical characteristics of the 12 individuals with *EYA4* variants. The onset age of hearing loss varied markedly from 5 to 61 years old; however, the onset of hearing loss in most cases was in the second decade or later. Mild to moderate hearing loss was observed in many cases, but two cases showed severe hearing loss. Asymmetric hearing loss was observed in two individuals (Family 1, 11). Audiometric configurations in these patients included low-frequency type in 6 ears, mid-frequency type in 2 ears, high-frequency type in 4 ears, and flat type in 12 ears. All individuals had noticed a progression in their hearing loss.

**Table 2:** Clinical features of affected family members with *EYA4* mutations found in this study.

Family No.	Nucleotide Change	Amino Acid Change	Sex	Domain	HL		Pure-tone audiometry			
					Onset (y)	Progression	Tested age (y)	PTA (R/L)	Severity (R/L)	Audiometric configuration (R/L)
Truncating variant										
1	c.222_223del	p.T74fs	M	V	61	Yes	64	35/52.5	mild/moderate	HF/LF
2	c.498delG	p.Q166fs	M	V	13	Yes	13	23.8/26.3	mild/mild	LF/LF
3	c.517C > T	p.Q173X	M	V	48	Yes	53	51.3/48.8	moderate/moderate	flat/flat
4	c.580 + 1G > A		F	V	45	Yes	47	52.5/56.3	moderate/moderate	flat/flat
5	c.910delC	p.P304fs	M	V	30	Yes	61	71.3/72.5	severe/severe	flat/flat
6	c.988C > T	p.Q330X	F	V	16	Yes	34	68.8/63.8	moderate/moderate	flat/flat
8	c.1177C > T	p.Q393X	M	E	26	Yes	36	61.3/63.8	moderate/moderate	flat/flat
11		CNV	F		25	Yes	51	75/57.5	severe/moderate	LF/HF
12		CNV	F		13	Yes	47	73.8/76.3	severe/severe	LF/LF
Non-truncating variant										
7	c.1109G > C	p.R370P	F	E	30	Yes	41	41.3/27.5	moderate/mild	MF/MF
9	c.1216G > C	p.G406R	M	E	5	Yes	77	51.3/63.8	moderate/moderate	flat/flat
10	c.1663G > C	p.A555P	M	E	25	Yes	37	55/53.8	moderate/moderate	HF/HF

Abbreviations: HL, hearing loss; HF, high-frequency hearing loss; MF, mid-frequency hearing loss; LF, low-frequency hearing loss; N/A, not available.

The article "Prevalence and clinical features of hearing loss caused by EYA4 variants" was published in 2020. Journal: Sci Rep.

### Analysis of hearing deterioration in the EYA4-associated hearing loss patients

To elucidate more precisely the type of hearing loss and rate of hearing deterioration, we collected the hearing thresholds of our patients. In addition, we also collected the hearing thresholds described in previous reports^5,16,20,27^. From our study results, we incorporated the hearing thresholds for 12 cases in this analysis (six cases considered to be unlikely causative variants were excluded from this analysis). We compared the hearing thresholds of patients with truncating variants to those with non-truncating variants (missense variants) including the patients in this study and previously reported cases (Fig. 2). As a result, the patients with truncating variants revealed a flat-type hearing loss that deteriorated in all frequencies, whereas the patients with non-truncating variants showed high-frequency hearing loss. We also analyzed the rate of hearing deterioration by using the patients in this study and previously reported case results (Fig. 3) and found that the average rate of progression in PTA was 0.63 dB/year (95%CI: 0.41–0.85 dB/year).

**Figure 2:** Audiometric configuration of *EYA4-*associated hearing loss. The left panel indicates the audiometric configuration of all of *EYA4-*associated HL. The center panel indicates the audiometric configuration of *EYA4-*associated HL with truncating variants. The right panel indicates the audiometric configuration of the *EYA4-*associated HL patients with non-truncating variants. This analysis was performed using the hearing thresholds from the 12 patients identified in this study and previously reported cases (n = 33). The blue line indicates 10–29 y. o. patients, the yellow line indicates 30–49 y. o. patients and the orange line indicates patients 50 y. o. or above.

The article "Prevalence and clinical features of hearing loss caused by EYA4 variants" was published in 2020. Journal: Sci Rep.

**Figure 3:** The estimated progression rate in PTA of *EYA4-*associated HL patients in this study and previous reports. The average progression rate in PTA was 0.63 dB/year.

## Discussion

In this report, we analyzed 1,334 ADNSHL patients and identified 12 candidate variants for *EYA4-*associated hearing loss. This is the largest population studied for *EYA4-*associated hearing loss to date. The prevalence of *EYA4-*associated hearing loss in ADNSHL was 0.90% (12/1,334 cases) in the Japanese population. This prevalence is slightly less than those of other ADNSHL genes such as *KCNQ4*, *TECTA*, *POU4F3*, and *WFS1*. *KCNQ4* is one of the most frequently observed responsible genes for ADNSHL in the Japanese population, and its prevalence is 6.6%^39^. Likewise, the prevalence of ADNSHL caused by *TECTA* variants is 2.9%, 2.7% for *POU4F3* variants, and 2.5% for *WFS1* variants^40–42^.

The responsible genes for ADNSHL differ among ethnic groups. For example, *KCNQ4* is the most frequent causative gene for ADNSHL in the Japanese population, whereas *TECTA* is the most frequent causative gene in the American population^43^. One plausible reason of this difference among populations is the effect of founder or recurrent mutations. Indeed, the variant of *KCNQ4*; c.211delC, which is commonly observed in Japanese ADNSHL patients, was reported to be caused by a founder effect^39^. Most of the *EYA4* variants found in this report were novel (we summarized the clinical features and identified variants of previous reports in Table 3) and the identified variants differed among patients. Only one variant (p.Q393X) was identified in a Korean patient^9^. According to this result, most of the *EYA4* variants are not recurrent. From these results, it appears difficult to find *EYA4* variants among autosomal dominant hereditary hearing loss patients by various genotyping analysis methods such as Invader assay or microarray, thus MPS is useful for identifying rare causative variants such as those in the *EYA4* gene in ADNSHL patients.

**Table 3:** Summary of the clinical features associated with *EYA4* mutations from previous studies.

Mutation type	Nucleotide Change	Exon/Intron	Amino Acid Change	Domain	Onset	Progression	Severity of HL	Audiometric Configuration	Family Origin	Reference
Missense or nonsense	c.152C > T	exon 4	p.S51F	Variable region	N/A	N/A	N/A	N/A	America	Sloan-Heggen, 2016^7^
	c.511G > C	exon 8	p.G171R	Variable region	6–50	Yes	mild to severe	flat, HF	China	Liu, 2015^5^
	c.863C > A	exon 11	p.S288X	Variable region	N/A N/A	N/A N/A	N/A moderate	N/A flat	Korea	Beak, 2012^8^ Kim, 2015^9^
	c.866C > T	exon 11	p.T289M	Variable region	N/A	N/A	N/A	N/A	America	Miszalski-Jamka, 2017^10^
	c.978C >G	exon 12	p.F326L	Variable region	N/A	N/A	N/A	N/A	Korea	Choi, 2013^11^
	c.1109G > A	exon 13	p.R370H	Eya domain	N/A	N/A	N/A	N/A	Philippines	Truong, 2019^12^
	c.1111G > A	exon 13	p.V371M	Eya domain	N/A	N/A	N/A	N/A	Belgium	Sommen, 2016^13^
	c.1154C > T	exon 13	p.S385L	Eya domain	N/A	N/A	N/A	N/A	Italy	Cesca, 2018^14^
	c.1177C > T	exon 13	p.Q393X	Eya domain	N/A	N/A	moderate	HF	Korea	Kim, 2015^9^
	c.1223G > A	exon 14	p.R408H	Eya domain	N/A	N/A	N/A	N/A	America	Miszalski-Jamka, 2017^14^
	c.1301T > A	exon 15	p.I434K	Eya domain	N/A	N/A	N/A	N/A	China	Tan, 2014^15^
	c.1643C > G	exon 18	p.T548R	Eya domain	19–37	Yes	mild to profound	flat, HF	China	Sun, 2015^16^
	c.1759C > T	exon 19	p.R587X	Eya domain	N/A	N/A	N/A	N/A	Belgium	Wayne, 2001^4^
	c.1810G > T	exon 19	p.G604C	Eya domain	N/A	N/A	N/A	N/A	Netherlands	Neveling, 2013^17^
	c.1834A > T	exon 19	p.K612X	Eya domain	N/A	N/A	mild to moderate	flat, HF	China	Hu, 2018^18^
Splicing	c.84-2A > G	intron 3			N/A	N/A	N/A	N/A	China	Chen, 2016^19^
	c.1282-12T > A	intron 14			6–30 s	Yes	moderate to severe	flat, HF	Australia	Hildebrand, 2007^20^
	c.1341-19T > A	intron 15			N/A	N/A	N/A	N/A	Germany	Vona, 2014^21^
	c.1739-1G > A	intron 18			50	N/A	N/A	N/A	America	Cirino, 2017^22^
Deletion	c.464delC	exon 8		Variable region	N/A	N/A	N/A	N/A	Sweden	Neveling, 2013^17^
	c.1194delT	exon 14	p.Met401Trpfs*3	Eya domain	20 s	Yes	moderate to severe	HF	Korea	Choi, 2016^23^
	c.1790delT	exon 19		Eya domain	35	Yes	moderate	flat	Japan	Iwasa, 2016^24^
Insertion	c.579_580insTACC	exon 8	p.Asp194Tyrfs*52	Variable region	N/A	N/A	N/A	N/A	Sweden	Frykholm, 2015^25^
	c.614dupA	exon 9		Variable region	N/A	N/A	N/A	N/A	China	Huang, 2015^26^
	c.1026_1027dupAA	exon 12		Variable region	N/A	N/A	N/A	N/A	America	Wayne, 2001^4^
	c.1048_1049dupAA	exon 12		Variable region	20s-40s	Yes	moderate to severe	flat, HF	America	Makishima, 2007^27^
	c.1115_1118dupTTGT	exon 13		Eya domain	N/A	N/A	N/A	N/A	Hungary	Pfister, 2002^28^
Gross deletion	10.4 Mb promoter and exon 1,2				N/A	N/A	N/A	N/A	Japan	Abe, 2009^29^
	4846 bp intron 10				N/A	N/A	N/A	N/A	America	Schönberger, 2005^30^
	9 Mb exon 4-20				N/A	N/A	N/A	N/A	Poland	Dutrannoy, 2009^31^

Abbreviations: HL, hearing loss; HF, high-frequency hearing loss; N/A, not available.

The article "Prevalence and clinical features of hearing loss caused by EYA4 variants" was published in 2020. Journal: Sci Rep.

In previous reports, the audiometric configuration for *EYA4-*associated hearing loss was a gradual high-frequency hearing loss or a flat-type hearing loss^44^. Further, no genotype-phenotype correlation was identified in previous reports. Kim *et al*. reported that no genotype-phenotype correlation existed for *EYA4-*associated hearing loss^9^. In their report, they analyzed only 87 ADNSHL patients, and identified only two patients carrying *EYA4* variants. In this study, we analyzed 1,334 ADNSHL patients, and identified 12 candidate *EYA4* variants. We also analyzed the detailed audiometric configurations of 12 patients identified in this study and previously reported cases and identified a genotype-phenotype correlation. High-frequency hearing loss was observed in patients with non-truncating *EYA4* variants, whereas flat-type hearing loss was observed in patients with truncating *EYA4* variants. In contrast, there were no significant differences in the severity of hearing loss among the different types of variants and/or variant locations (domain).

We also analyzed the rate of hearing deterioration in *EYA4-*associated hearing loss patients identified in this study and previously reported cases. The rate of progression of hearing loss caused by *EYA4* was considered to be 0.63 dB/year (95%CI: 0.41–0.85 dB/year). In previous reports on ADSNHL hearing loss, the progression rate for the *POU4F3* gene was 0.5–0.9 dB/year^41^, that for *MYO6* was 2.0 dB/year^45^, and that for *ACTG1* was 2.0–6.0 dB/year^46^, and the results in this study suggests that the rate of hearing loss progression caused by *EYA4* may be relatively mild.

In this study, we identified nine truncating variants including two *EYA4* copy number loss cases. Thus, we speculated that the mechanism of *EYA4-*associated hearing loss was haploinsufficiency. In the gnomAD database (https://gnomad.broadinstitute.org/gene/ENSG00000112319), a non-negligible number of truncating variants were identified in large control populations. The probability of a loss of function intolerant score (pLI score) was 0.05. This low score may mean the loss of function in this gene is tolerant and without pathogenicity. However, most of the loss of function variants were located in specific exons that only included some splicing variants and were seldom observed in other exons (Fig. 4). From these observations, we hypothesized that these specific isoforms may not be expressed in the inner ear or may not play an important role in hearing function. It is unknown which isoforms are expressed in the human inner ear. As another hypothesized mechanism, loss of function variants in the gnomAD database were accumulated in the second to last exon, and these variants might not trigger nonsense-mediated mRNA decay. Thus, these loss of function variants may not cause hearing loss. The identified truncating variants, except for c.1790delT, were located in the exons which were included in all isoforms carried. The prevalence of loss of function variants in the *EYA4* gene was 19 among about 250,000 alleles in the gnomAD database, but 9 among 2,672 alleles in this study. The summarized odds ratio between our hearing loss cohort vs. gnomAD was 44.469 (95%CI: 20.495–96.490). This result also supports haploinsufficiency as the mechanism underlying *EYA4-*associated hearing loss. The patient who carried c.1790delT, located in specific exons (truncating variants accumulated in the exon in gnomAD) suffers from an enlarged vestibular aqueduct, and this phenotype was not matched with hearing loss caused by *EYA4* mutations. For these reasons, we classified this variant (c.1790delT) as “unlikely causative”.

The article "Prevalence and clinical features of hearing loss caused by EYA4 variants" was published in 2020. Journal: Sci Rep.

**Figure 4:** The location of truncating variants identified in this study, previous reports and the genomAD database. The schema shows alternative splicing variants of the *EYA4* gene. Black boxes indicate exons present in each transcript variant and black lines indicate introns. Blue arrows indicate truncating variants identified in this study. Green arrows indicate truncating variants identified in previous reports. Red arrows indicate truncating variants in the genomAD database.

In conclusion, we performed MPS analysis of large cohort of 1,334 ADNSHL patients and successfully identified 12 novel and promising pathogenic variants. Based on this, we estimated the incidence of *EYA4-*associated hearing loss was 0.90% in Japanese families with autosomal dominant hearing loss. The audiometric configuration of truncating variants tended to exhibit flat-type, whereas that of non-truncating variants tended to be high-frequency hearing loss, suggesting a novel genotype-phenotype correlation in DFNA10.
